# Emergency Nursing Countermeasures and Experience of Patients with Primary Liver Cancer Nodule Rupture and Hemorrhage

**DOI:** 10.1155/2022/2744007

**Published:** 2022-07-05

**Authors:** Yanyun Qing, Juan Yang, Yanli Gu

**Affiliations:** The Nanhua Affiliated Hospital, Department of First Oncology, Hengyang Medical School, Universitity of South China, Hengyang, Hunan 421002, China

## Abstract

**Objective:**

To explore the emergency nursing countermeasures and nursing experience of patients with primary liver cancer nodule rupture and hemorrhage.

**Methods:**

30 patients with primary liver cancer nodule rupture and hemorrhage treated in our hospital since January 2020 after the implementation of emergency nursing countermeasures were selected as the observation group, and another 30 patients with primary liver cancer nodule rupture and hemorrhage treated in our hospital before January 2020 were selected as the control group. The control group received basic nursing intervention, while the observation group received emergency nursing measures. The hemoglobin level, blood oxygen saturation monitoring value, and partial pressure of oxygen of patients with hemorrhagic shock due to nodular rupture of primary liver cancer were compared between the two groups at admission and after nursing care. All indexes of patients during the perioperative period were recorded. The incidence of complications, mortality, and nursing satisfaction rates of the patients' families were compared between the two groups.

**Results:**

After nursing care, the observation group's patients' hemoglobin level, blood oxygen saturation monitoring value, and partial pressure of oxygen were higher than those of the control group's patients (*P* < 0.05). The intraoperative bleeding volume, shock correction time, and discharge time of patients in the observation group were lower than those of patients in the control group (*P* < 0.05). The incidence of complications and mortality in the observation group was significantly lower than those in the control group (*P* < 0.05). The nursing satisfaction rate of patients in the observation group was higher than that of the control group (*P* < 0.05).

**Conclusion:**

The results of emergency nursing intervention in patients with primary liver cancer rupture and hemorrhage are reliable, which can significantly improve perioperative indicators of patients, reduce complications and mortality, improve nursing satisfaction, and effectively shorten the hospital stay of patients.

## 1. Introduction

Primary liver cancer is the fifth largest malignant tumor in the world, and its incidence is increasing year by year. It is estimated that, by 2025, more than one million new cases of liver cancer will be discovered every year [1–3]. There is a large population with liver cancer in China. Fifty-five percent of the world's liver cancer patients are in China. Primary liver cancer has become the second leading cause of cancer death in China. Most of the patients with early primary liver cancer have no obvious symptoms. 85% to 90% of the patients were found to be in the middle and late stages [4–6]. Some patients were first discovered when they were admitted to the hospital because of an acute abdomen rupture caused by liver cancer. Spontaneous rupture and hemorrhage of primary liver cancer nodules are one of the four major factors of death in patients with liver cancer, and its incidence rate is 7%–20%. The rupture of liver cancer can easily cause massive hemorrhage, leading to local tissue ischemia and hypoxia, bacterial translocation, secondary infection, severe hemorrhagic shock, or even septic shock in a short time. The condition is critical and complicated, and the prognosis is poor, which endangers the life of the patient [7, 8]. Hemorrhage due to a rupture of nodules of primary liver cancer is a serious complication, and its treatment and nursing are difficult. At present, emergency interventional embolization is commonly used clinically to treat primary liver cancer with nodular rupture and hemorrhage, which can effectively control the progression of the disease and prolong the survival time of patients [9, 10]. However, it is very important to treat the ruptured primary liver cancer nodules with emergency interventional embolization, and there are many postoperative complications. Therefore, it is particularly important to take timely and effective nursing intervention on primary liver cancer nodule rupture and hemorrhage, which can reduce postoperative complications and improve the quality of life of patients [11, 12]. This study compared the perioperative nursing effects of patients with nodular rupture and hemorrhage of primary liver cancer before and after the implementation of emergency nursing measures in our hospital and summarized the experience and value of emergency nursing measures. The results are now reported as follows.

## 2. Data and Methods

### 2.1. General Information

30 patients with primary liver cancer nodules rupture and hemorrhage who have been treated in our hospital since January 2020 after the implementation of emergency nursing countermeasures were selected as the observation group, including 21 males and 9 females, aged 40–65 years. In addition, 30 patients who were admitted to our hospital before January 2020 with nodular rupture and hemorrhage of primary liver cancer were selected as the control group, including 22 males and 8 females, aged 42–68 years. Inclusion criteria were as follows: all patients received a clinical physical examination, blood biochemistry, and imaging examinations, which were consistent with the diagnosis of primary liver cancer; all patients had a sudden and severe upper abdominal pain and blood pressure drop, accompanied by symptoms and signs of hemorrhagic shock, such as pale complexion, cold limbs, tachypnea, and syncope; all patients had diagnostic paracentesis to draw blood samples or red hemorrhagic ascites; all patients' clinical data were intact. Exclusion criteria were as follows: early death patients; patients who are delirious and unable to cooperate with the treatment; lack of clinical data; patients who failed to follow-up or were transferred to a hospital for treatment.

### 2.2. Research Methods

The control group received basic nursing intervention, and the patients were sent to the emergency room quickly. The patient's lower limbs were raised by 30 degrees, lying on his back, and his head was tilted to one side. A venous access was established, and fluid replacement was performed to correct the shock. Patients were treated with routine symptomatic treatment, such as hemostasis, volume expansion, and blood transfusion.

The observation group took emergency nursing measures. Comprehensive emergency care was given to patients from various aspects.

Preoperative nursing was as follows:

(1). Two or more venous pathways were established. First of all, deep vein intubation (internal jugular vein or subclavian vein puncture) was considered to be beneficial to rapid blood transfusion and expansion, and correction of shock. At the same time, central venous pressure was monitored to regulate infusion volume and infusion speed. In addition, a venous indwelling needle was retained through a peripheral venous puncture, which can be used for the infusion of other therapeutic drugs.
(2). Patients with liver cancer rupture bleeding with shock, which can cause organ hypoperfusion, timely expansion to maintain effective circulation blood volume of important organs, and correction of shock is the focus of treatment. A colloid solution (red blood cells and plasma) shall be infused first when rehydrating, and the sequence of rehydration shall be arranged reasonably, so as to replenish blood volume in time and improve the heartbeat. Hemostatic drugs (somatostatin) shall be taken into consideration, and water, electrolyte, and acid-base balance disorders shall be corrected simultaneously. Nurses need to understand the role of drugs, side effects, and incompatibility.
(3). patients with liver cancer rupture and bleeding according to the situation of the blood loss to input a large amount of whole blood, the nurse need to strictly implement the system of blood transfusion check and closely observe the presence of blood transfusion reaction.
(4). patients with liver cancer rupture bleeding hematemesis, easy to cause aspiration and cause suffocation, nursing should be timely cleaning respiratory secretions and vomit, paying attention to keep the patient's respiratory tract patency.
(5). Closely observe the patient's vital signs, every 15 min measurement of patients with blood pressure, pulse, respiration, central venous pressure, and continuous ECG monitoring. Observe the patient's consciousness changes and skin mucosa (color changes of face and lips) to determine the peripheral circulation. The urine volume (hourly urine volume and 24 h urine volume) and abdominal condition (abdominal pain, abdominal distension, and abdominal muscle tension) were observed.
(6). Ready for emergency surgery. We should carry out perfect various preoperative preparations as soon as possible, including skin preparation, urinary catheter insertion, blood typing, coagulation time determination, and biochemical tests.
(7). patients with liver cancer rupture bleeding, consciousness is clear, the spirit is hard to bear, easy to appear fearful, and to have an agitated state of mind. We should pay attention to the transfer of patients' bad emotions, do a good job in psychological counseling, give them spiritual support and encouragement, through counseling, and encourage them to adjust their emotions through counseling. Doing a good job in all kinds of treatment and life care and concentrating on all kinds of treatment and care as much as possible, so as to reduce the turnover and unnecessary pain of patients. Relying on skilled technology and rigorous work style to win the trust of patients, patients can actively cooperate with treatment and care..

Postoperative nursing was as follows:

(1). Closely monitor the vital signs of patients after operation and accurately record the amount of fluid in and out. Do a good job in surgical handover, give oxygen using a nasal catheter, instruct patients to stay in bed absolutely, reduce physical energy consumption, increase liver blood flow, and promote liver function recovery. Check whether the dressing at the puncture point of the femoral artery in the groin is dry, whether there is bleeding and swelling and whether the dorsalis pedis artery beats.
(2). Maintain effective ventilation in the ward, and conduct disinfection and isolation management on the ward environment, including air disinfection. The ground, walls, and surfaces of objects are cleaned by the wet method to reduce air flow; fixed family escort and strict restrictions on personnel visits; medical staff should wash their hands carefully, wear masks, and strictly implement aseptic operation procedures before contacting patients.
(3). Observe the patient's fever degree and state, record the temperature, and draw the temperature change curve. When the body temperature is less than 38.5°C, the patient can temporarily stop taking medicine, and physical antipyretic methods such as cold compress on the head and bathing can be given. When the body temperature is above 38.5°C, appropriate antipyretic and analgesic drugs can be selected according to the doctor's advice, and patients should be instructed to drink plenty of water to help reduce fever and prevent excessive sweating from collapse.
(4). Postoperative pain in the liver area of the patient is mainly caused by the blockage and spasm of the responsible blood vessel by the embolic material, which causes acute ischemia of the target organ and the vascular tissue around the tumor, resulting in pain. The causes of pain to patients and their families are explained to relieve their worries. If the pain is severe, accompanied by systemic symptoms, those with peritoneal irritation are likely to bleed again.
(5). Improve a variety of nursing documents, records of intensive care were made, not only for the diagnosis and treatment to provide reliable medical data and take the corresponding treatment measures but also to guarantee the means of nursing occupational safety.

The hemoglobin level, blood oxygen saturation monitoring value, and partial pressure of oxygen at the time of admission and after nursing care of patients with hemorrhagic shock due to nodular rupture of primary liver cancer were compared between the two groups. Perioperative indicators of the patients were recorded, such as operation time, intraoperative bleeding volume, time to correct shock, and time to cure and discharge. The incidence of complications and mortality were compared between the two groups.

### 2.3. Statistical Methods

SPSS22.0 software was used for processing. The measurement data were expressed as mean standard deviation ($\bar{x}\pm s$), and the *t*-test was used for pairwise comparison. Enumeration data were expressed as (%), and the *χ*^2^ test was used for enumeration data. The test level was *α* = 0.05, and *P* < 0.05 indicated that the difference was statistically significant.

## 3. Results

### 3.1. Comparison of General Data between the Two Groups

There were no significant differences in gender, age, Child-Pugh classification, and clinical manifestations between the two groups (*P* > 0.05) as shown in Table 1.

### 3.2. Comparison of Hemoglobin Level, Blood Oxygen Saturation Monitoring Value, and Partial Pressure of Oxygen between the Two Groups

There was no significant difference in the hemoglobin level, blood oxygen saturation monitored value, and oxygen partial pressure between the two groups at the time of admission (*P* > 0.05). After nursing, the hemoglobin level, blood oxygen saturation monitoring value, and partial pressure of oxygen in the observation group were higher than those in the control group, and the differences were statistically significant (*P* < 0.05) as shown in Figures 1–3.

### 3.3. Comparison of Perioperative Indicators between the Two Groups

There was no significant difference in operation time between the two groups (*P* > 0.05). The intraoperative bleeding volume, shock correction time, and discharge time of patients in the observation group were lower than those of patients in the control group, and the differences were statistically significant (*P* < 0.05), as shown in Figures 4–7.

### 3.4. Comparison of Complication, Incidence, and Mortality between the Two Groups

The incidence of complications and mortality in the observation group was significantly lower than those in the control group, and the differences were statistically significant (*P* < 0.05), as shown in Figure 8.

### 3.5. Comparison of the Nursing Satisfaction Rate between the Two Groups

The nursing satisfaction rate of patients of the observation group was higher than that of the control group, and the differences were statistically significant (*P* < 0.05), as shown in Figure 9.

## 4. Discussion

Rupture and hemorrhage of primary liver cancer nodules is a serious complication of primary liver cancer nodules with a high mortality rate [13, 14]. Our patient has an acute onset, which is sudden and fierce. His condition is changing rapidly and he often suffers from hemorrhagic shock. In case of rupture and bleeding, we should give priority to controlling bleeding and saving the patients' life, observe the patients' condition dynamically, adjust the treatment and nursing measures in time, and make preoperative prevention and nursing. Careful observation of the condition, early detection of the changes of the condition, and quick and effective rescue and nursing measures are the key to successful rescue [15–17].

This research shows that, after nursing, the patients in the observation group were significantly better than those in the control group in hemoglobin level, oxygen saturation monitored value, and partial pressure of oxygen. Correction of the shock not only creates conditions for the operation but also reduces the risk of operation and postoperative complications. Therefore, preoperative antishock therapy is the key to the treatment of rupture and hemorrhage of liver cancer nodules, and it is also a test of the medical staff's first aid ability [18, 19]. The study also showed that the patients in the observation group had a lower intraoperative bleeding volume, shock correction time, and discharge time than those in the control group. It indicated that the adoption of emergency nursing countermeasures, which improved the quality of nursing care as a whole, actively cooperated with the correction of shock, and preparation for emergency surgery at the same time, had become the key to rescue the rupture and hemorrhage of liver cancer nodules [20, 21].

Emergency nursing countermeasures included rapid establishment of infusion channels, reasonable selection of infusion sequence, dynamic observation of the condition, preparation for emergency surgery, and psychological intervention. Unlike elective liver cancer surgery, the nursing care of patients with ruptured liver cancer nodules in an emergency requires all measures to be based on the principles of stopping the bleeding and saving lives. The nursing procedure is composed of many links, and the nursing risk runs through many links, such as cooperation with rescue and nursing operations. Only by paying attention to the detailed management of all aspects of nursing, making the work carefully, doing well, and controlling the quality of the link, can we improve the cure rate of patients and the success rate of rescuing critically ill patients, avoiding nursing risks and ensuring nursing safety [22–24]. Finally, the complications and mortality between the two groups showed that the incidence of complications and mortality in patients of the observation group was significantly lower than that of the control group. Patients with primary liver cancer nodules rupture and hemorrhage have an urgent disease onset. When patients are admitted to the hospital, the nurses carry out a comprehensive understanding and evaluation of the patients' condition, dynamically observe the changes in the patients' vital signs and consciousness, identify potential and possible risk factors, and complete the emergency and preoperative care procedures, which are conducive to reducing the mortality rate of patients [8, 25, 26].

When facing liver cancer for the first time, most patients are still conscious and overwhelmed, showing fear and despair. At this point, the nursing work should pay attention to transferring the patients' bad emotions and do a good job of psychological counseling. It is necessary to understand the patients' personality and psychology, apply the concept of psychological nursing, provide respect and care for patients, give the patient spiritual support and encouragement, and adjust the patients' emotions through persuasion and comfort. At the same time in nursing, relying on skilled technology and a rigorous work style to obtain the patients' trust, so that patients can actively cooperate with the treatment and nursing [27, 28]. The results showed that the nursing satisfaction rate of patients in the observation group was higher than that of patients in the control group. It indicated that the adoption of emergency nursing countermeasures had good effects on the improvement of nursing satisfaction.

In summary, the emergency nursing countermeasures in patients with primary liver cancer nodules rupture bleeding application effect is good and can significantly improve the perioperative indicators of patients, reduce complications and mortality, improve nursing satisfaction, and effectively shorten the hospital stay of patients.

## Figures and Tables

**Figure 1:** Comparison of the hemoglobin level between the two groups. Note: compared with the control group, ^*∗*^*P* < 0.05.

**Figure 2:** Comparison of oxyhemoglobin saturation monitoring between the two groups. Note: compared with the control group, ^*∗*^*P* < 0.05.

**Figure 3:** Comparison of oxygen partial pressure between the two groups. Note: compared with the control group, ^*∗*^*P* < 0.05.

**Figure 4:** Comparison of the operation time between the two groups.

**Figure 5:** Comparison of the intraoperative bleeding volume between the two groups. Note: compared with the control group, ^*∗*^*P* < 0.05.

**Figure 6:** Comparison of the shock correction time between the two groups. Note: compared with the control group, ^*∗*^*P* < 0.05.

**Figure 7:** Comparison of the discharge time between the two groups. Note: compared with the control group, ^*∗*^*P* < 0.05.

**Figure 8:** Comparison of complication incidence and mortality between the two groups. Note: compared with the control group, ^*∗*^*P* < 0.05.

**Figure 9:** Comparison of the nursing satisfaction rate between the two groups. Note: compared with the control group, ^*∗*^*P* < 0.05.

**Table 1:** Comparison of general data between the two groups.

*Group*	*N*	*Male/female*	*Age (years)*	*Child–Pugh classification*		*AFP* *>* *200 μg/L*
				*Class II*	*Class III*	

Control group	30	22/8	52.96 ± 3.84	14	16	21
Observation group	30	21/9	51.83 ± 3.17	13	17	20
* t/χ* ^2^ *value*		0.082	1.243	0.067		0.077
*Pvalue*		0.774	0.219	0.795		0.781

*Group*	*N*	*Clinical picture*				
		*Jaundice*	*Palpitate*	*Abdominal tenderness*	*Hepatomegaly*	*Right upper quadrant palpable mass*

Control group	30	18	15	27	30	15
Observation group	30	19	14	28	29	16
* χ* ^2^ *value*				0.124		
*Pvalue*				0.998		

## Data Availability

The data can be obtained from the author upon reasonable request.
